RETRACTED

# The Influence of Teachers' Management Efficiency and Motivation on College Students' Academic Achievement under Sustainable Innovation and the Cognition of Social Responsibility after Employment

**DOI:** 10.1155/2022/1663120

**Published:** 2022-08-25

**Authors:** Chang Tan, Lianyun Yi, Aziz Haider, Liew Kwen, Rahman Mamnoon, Keqing Li, Min Liu

**Affiliations:** ^1^Southwest University, Beibei, China; ^2^Chongqing University of Education, Chongqing, China; ^3^Hainan Normal University, Haikou, China; ^4^University of Tikrit, Tikrit, Iraq; ^5^College of Information Science and Engineering, Management and Science University, Shah Alam, Malaysia; ^6^National University of Sciences and Technology, Islamabad, Pakistan; ^7^City University of Hong Kong, SAR, Hong Kong, China; ^8^Shanxi University, Taiyuan, China

## Abstract

Teachers' management effectiveness can reflect the comprehensive ability and effective evaluation of the teaching management objectives of the school and can also reflect the effectiveness management of the school to a certain extent. In the environment of sustainable and innovative development, the rapid development of education has made improving the management efficiency and motivation of university teachers became the key direction of university management. In order to study the impact of teachers' management efficacy and motivation on college students' academic achievement and postemployment social responsibility cognition under sustainable innovation, this study compares the impact of teachers in different periods on students and analyzes the changes of teachers in different periods on students. Finally, it is concluded that teachers' management efficiency and motivation under sustainable innovation can promote students' employment achievement and social responsibility cognition, improve the teaching quality of colleges and universities, and provide high-quality talents for the country. The educational concept of sustainable innovation is conducive to improving teachers' independent innovation and realizing the educational function of cultivating students' personalized development in colleges and universities.

## 1. Introduction

Colleges and universities are educational bases for the country to cultivate talents for the society. Teachers are the main body of teaching management. The management of teachers directly affects the teaching quality of colleges and universities. Xia proposed that teaching management efficiency is a comprehensive ability for colleges and universities to achieve teaching management objectives, which is mainly based on the effective utilization of various resources, and also reflects the school efficiency to a certain extent. The rapid development of education makes the improvement of teaching management efficiency play an important role in the teaching effect of colleges and universities and the employment prospect of students [1]. In this regard, Pan pointed out that the problems encountered in the current teaching work in colleges and universities and reflective teaching guidance are required to strengthen teachers' functions, strengthen management efficiency, and innovate work ideas [2]. The improvement of teachers' skills directly affects students' studies. Jiang pointed out that the management efficiency of colleges and universities directly affects the future development direction of colleges and universities. It is the basis of teaching and has a direct impact on the improvement of teaching quality. The curriculum management efficiency of colleges and universities is mainly divided into higher vocational college background, teaching ability, service awareness, teachers, teaching environment, basic equipment, curriculum guidance, teaching mode, working mode, and moral cultivation [3]. With the improvement of all aspects of the school, teachers' teaching methods have also improved. Zhou and Zhengshuchao showed that teachers' working ability is a necessary comprehensive ability for teachers to complete tasks, which directly affects the efficiency of teachers' work and the efficiency of teaching management. The survey found that college teachers' working ability is generally high, and their teaching ability is also good; in addition, income, gender, school level, professional title, educational background, and other characteristics have a significant impact on the level of teachers' working ability, which is directly related to the management of teaching effectiveness [4]. Excellent teachers tend to develop in many ways, which is very beneficial to students. Wuxiaohuan pointed out that university management has a direct impact on the work of teaching and scientific research in colleges and universities and is related to the further development of colleges and universities. At present, there are still many problems in university management. Take the party's mass line as the guiding ideology, implement the party's mass line, and improve university management [5]. Teachers should set up the basic concept of taking students as the basic idea, enhance service awareness, work actively, encourage innovation, improve students' enthusiasm, and recognize their self-worth. Zhang pointed out that college students are the talent reserve of the society, and education is an inevitable requirement to promote social development and progress of the times [6]. Colleges and universities should shoulder the responsibility of innovation and cultivate comprehensive talents. Dingyi proposed that, in the rapid development of social economy and the continuous improvement of people's living standards, in order to improve teaching methods and change teaching modes, colleges and universities should shoulder their own responsibilities and make contributions to improving students' employability [7]. The change of teaching mode and the acquisition of various knowledge have enabled students to find their own position. Liuzhenzhong pointed out that students have weak sense of responsibility and unclear responsibility goals in the process of employment. Through the identification of different responsibilities of the government, universities, teachers, students, and society in the process of college students' employment, we can clarify the school running goals and actively make career planning for college students. Thus, actively constructing the employment sharing mechanism for college students can promote the full and effective employment of college students [8]. In this regard, Kuang and Guopengyi proposed that the sustainable development of society cannot be separated from sustainable innovation education. Sustainable innovation education is actually internal education. Based on the education of complete personality, we should improve the educational concept, combine the current situation of college students' study and life, constantly innovate educational methods and optimize the educational environment, enhance the comprehensiveness of college education, and realize sustainable innovation education [9]. Through the research on the impact of teachers' management efficacy and motivation on college students' academic achievement and the cognition of social responsibility after employment under sustainable innovation, this study understands that the most important work for colleges and universities to improve efficiency management is to improve teachers' self-efficacy management and teaching results, improve students' comprehensive performance, recognize their own advantages, and integrate the realistic sense of responsibility into social life, that is, being a useful person to the society.

RETRACTED

## 2. The Influence of Professional Title on Teachers' Achievement Motivation in Colleges and Universities

Professional title is an important variable that affects the management efficiency and motivation of teachers in colleges and universities. Different people have different views on professional title, which will also have different effects on the management efficiency and motivation of teachers. When teachers pay more attention to the honor and status brought by professional titles, the more urgent the pursuit of professional titles, the higher the management efficiency and the stronger the motivation. The professional titles of colleges and universities include teaching assistants, lecturers, associate professors, and professors. By comparing the impact of professional titles on the management effectiveness and motivation of traditional teachers and innovative teachers, the results are shown in Table 1.

In Table 1, the motivations of teaching assistants, lecturers, associate professors, and professors in traditional teaching are 79%, 85%, 88%, and 86%, respectively, and the motivations in innovative teaching are 88%, 95%, 92%, and 94%, respectively. The motivation level of teachers after innovation is slightly higher than that before innovation. Convert Table 1 data into a visual diagram, as shown in Figure 1.

It can be concluded from Figure 1 that the evaluation of professional titles has a certain relationship with teachers' wages and social status. Whether before or after innovation, the evaluation of professional titles has a great impact on teachers' achievement motivation. The professional title evaluation after the reform and innovation can stimulate the enthusiasm, initiative, and creativity of college teachers and better develop modern education with Chinese characteristics, and to a certain extent, it will also drive the development of students in all aspects. The evaluation of teachers' professional titles after innovation is also an important measure for teachers' management efficiency and motivation. It can further stimulate the teaching quality of colleges and universities, improve various assessment and evaluation mechanisms of teachers, and continuously stimulate teachers' vitality and innovation.

## 3. The Influence of Educational Background on Teachers' Professionalism

Academic qualifications also have a certain impact on the professionalism of teachers in colleges and universities. Teachers with different educational background have different professional identity, professional ethics, professional knowledge, and professional ability. If teachers' professional ability is strong, their management efficiency will be correspondingly high, and their motivation will be strong. Under the background of sustainable innovation, teachers will also keep pace with the times for teaching and educating people.  Table 2 and Figure 2 are obtained by comparing various aspects of college teachers with different academic qualifications under sustainable innovation.

From Table 2 and Figure 2, it can be seen that the professionalism of teachers with graduate degrees in the four aspects of professional identity, professional ethics, professional knowledge, and professional ability is 95%, 93%, 97%, and 92%, respectively, which is higher than the other two degrees, while the professionalism of undergraduates is slightly higher than that of junior colleges. It can be seen that the strengthening of teachers' professional ability can not only enhance their own management efficiency and motivation, but also improve students' cognition and interest in their major and enhance students' learning motivation and academic pursuit.

RETRACTED

## 4. Analysis on the Circulation Characteristics of Teachers' Management Efficiency under Innovation

The development of scientific research and social progress have made new breakthroughs in various industries under the conditions of innovation. Innovation idea means that an enterprise or individual breaks the convention, breaks through the current situation, dares to be the first, dares to challenge the future, breaks the mindset, and seeks a new realm. The premise of innovation is dissatisfaction with the current situation. At the same time, innovation is based on the correct grasp of the market law and the development prospect of the industry. It is also widely used in the field of education. The formation and development of teachers' efficacy will naturally be influenced by teachers' actual teaching experience, that is, mastering experience, and observing the experience gained by model teachers' teaching, that is, substituting experience, social persuasion, and teachers' own emotions. At the same time, teachers' efficacy will also be affected by the students and classes taught, the school environment and cultural atmosphere, and the collective efficacy of school teachers. Based on their own knowledge, ability, and skills, teachers engage in practical educational and teaching activities to achieve success, which is the basic condition for improving teachers' effectiveness. The success or failure experience of educational and teaching practice has the most important impact on the formation and development of teachers' effectiveness.

Therefore, the teacher management effectiveness is analyzed according to the cycle characteristics, and the relationship between them is shown in Figure 3.

As shown in Figure 3, emotional arousal, language persuasion, substituting experience, mastering experience, and new efficacy information, through their own cognitive processing process, form two different analysis results: teaching task analysis and personal teaching ability evaluation. The two are decomposed and analyzed through teachers' functional efficacy. The analysis of teaching tasks will affect the establishment of general teaching effectiveness, and the evaluation of individual teaching ability is the basis for the formation and development of individual teaching effectiveness.

RETRACTED

## 5. Research and Analysis on the Formation Stage and Development of Teachers' Teaching Ability under Sustainable Innovation

With the increasing impact of science, economy, technology, and environment on various fields of human life, the requirements of the state and society for teachers are also becoming higher and higher. A qualified teacher needs to have general cultural knowledge, specialized knowledge of the disciplines he teaches, knowledge of educational disciplines, and basic education and teaching ability. The high requirements urge teachers and relevant educational institutions to pay attention to teachers' professional level. Teachers' professional development has become a hot spot in the educational field in recent years. Improve their professional teaching ability according to their basic ability, so as to develop the performance with ontology core ability.  Figure 4 is drawn according to the relationship between them.

As shown in Figure 4, the pedagogical theory, the professional knowledge of the ontology, and the individual quality of teachers form the general ability. The general ability is divided into the professional quality of higher vocational teachers, the function of higher vocational teaching knowledge, and cognitive ability. These three basic abilities are upgraded to special abilities. After being promoted to a special ability, the implementation ability, management ability, and monitoring ability of higher vocational teaching have been developed and innovated. Finally, it is the core competence of teachers' profession. The teaching development idiosyncrasy and teaching philosophy literacy have been practically applied and practiced on the basis of innovation. The improvement of individual basic ability and the combination of professional teaching ability have certain foundation for the core ability of ontology. Therefore, the teacher management efficiency under the innovation not only has a certain good effect on the development of professional teaching, but also on the society itself.

## 6. Analysis on the Influence of Management Efficiency and Motivation on College Students' Academic Achievement in Different Periods

### 6.1. Comparison of Teacher Management Efficacy on Academic Achievement of College Students in Different Periods

Teachers' management effectiveness is mainly affected by external environment and teachers' subjective factors. The external environment mainly includes students' characteristics, school background, and interpersonal communication. Teachers' subjective factors mainly include teachers' experience, self-cognition, and teaching ability. When external factors and subjective factors change, teachers' management effectiveness will also change, and the impact on students' academic achievement is also different. The comparative study of teacher management effectiveness in different periods is as follows.

RETRACTED

In Table 3, through the research on the teaching management effectiveness of teachers in different periods, the traditional teachers' curriculum learning, interpersonal communication, ability training, and academic evaluation are 40, 58, 67, and 43%, respectively, while those of teachers under sustainable innovation are 88, 85, 91, and 93%, respectively. The improvement of teachers' teaching management efficiency will have a profound impact on students' behavior norms and self-efficacy and can also correctly guide students' employment.

In order to observe the difference between the two more conveniently, the above data is transformed into a visual comparison diagram, as shown in Figure 5.

As can be seen from Figure 5, the effect of teacher management efficacy on students' academic achievement under the background of sustainable innovation is better than that of traditional teacher management efficacy on students' academic achievement. Therefore, it can be considered that, in the context of sustainable innovation, teacher management effectiveness plays a promoting role in the impact of students' academic achievement.

### 6.2. Comparison of Teacher Motivation on College Students' Academic Achievement in Different Periods

Teaching motivation can be divided into internal motivation and external motivation. The internal motivation includes interest in teaching, professional responsibility, and satisfaction of self-achievement. The external motivation includes school's encouragement to teachers and external affirmation to teaching. Teachers' teaching motivation has a direct impact on teachers' teaching work. When teachers' teaching motivation is weak, their enthusiasm for teaching will be low, and students' academic achievement will be low. When the teaching motivation is strong, the teaching enthusiasm will increase correspondingly, and the students' academic achievements will also improve relatively. In order to study and analyze the impact of teachers' motivation on students' academic achievement in different periods, traditional teachers and teachers under sustainable innovation are compared.  Table 4 is as follows.

In Table 4, through the analysis of the data on the impact of the above two different periods on students' academic achievement, it can be clearly seen that, among teachers' motivations such as achievement motivation, responsibility motivation, education guarantee, and teaching level pursuit, the influence of teachers under sustainable innovation on students' academic achievement is 89%, 94%, 81%, and 92%, respectively, which is significantly higher than that of traditional teachers. Teachers under sustainable innovation have significantly improved students' academic achievement compared with traditional teachers, which is more conducive to college students' academic planning and targeted employment choices, and better ensure the achievement development in the later period.

RETRACTED

The comparison data of teacher motivation in two different periods are visualized as shown in Figure 6.

Figure 6 shows the data comparison between traditional teachers and teachers' academic achievements of college students under sustainable innovation. The comparison results show that innovative teachers have higher academic achievements than students. It can be considered that teachers' motivation under continuous innovation is more conducive to improve students' academic achievement.

## 7. Analysis of Teachers' Management Efficacy and Motivation on Students' Postemployment Social Responsibility Cognition in Different Periods

### 7.1. Comparison of Teachers' Management Effectiveness on Students' Postemployment Responsibility Cognition in Different Periods

With the rapid development of economy, the society has made continuous innovation and progress. In the field of education, the management efficiency of teachers is also constantly improving. The efficiency concept of teacher management refers to the management behavior of school administrators on teachers, focusing on the cultivation of teachers' sense of education and teaching efficacy. Through the cultivation of teachers' sense of self-efficacy, teachers' enthusiasm for work is stimulated, and teachers are encouraged to comprehensively improve their working ability in the active subject education practice efficiency and professionalism is a kind of teacher management concept. The social responsibility of students after employment refers to the responsibility of an organization to the society. An organization should operate and manage in a way conducive to society. Social responsibility usually refers to the social obligations undertaken by the organization higher than its own goals. Management efficiency goes beyond the obligation of law and economy to the organization. Social responsibility is the requirement of organizational management ethics, and it is a voluntary act of the organization out of obligation.

In order to better understand the management effectiveness under tradition and innovation and analyze teachers' sense of efficacy, knowledge management, social responsibility cognition, ideals, and beliefs, Table 5 is drawn according to the analyzed data values.

RETRACTED

In Table 5, it is clear that the data values of teacher efficacy, knowledge management, social responsibility cognition, ideals, and beliefs in traditional management efficacy are all around 50%; on the contrary, the data values of innovation management efficacy are all above 50%, which is significant.

In order to observe the contrast between the two more intuitively, a viewable Figure 7 is drawn according to the data values in Table 5.

As shown in Figure 7, comparing the data values of various factors in the traditional management efficiency and innovation pipeline efficiency, we can see that the data values under innovation have advantages, and the data values are relatively high, while the data values of the traditional management efficiency are generally not high, and there is no significant contrast. Therefore, innovation can not only improve the change of data value, but also lay a foundation for the later improvement of efficiency.

### 7.2. Analysis of Teachers' Motivation on Students' Social Responsibility after Employment in Different Periods

Teacher motivation refers to the undetermined psychological tendency of teachers' work motivation to meet teachers' needs and promote teachers to achieve the specific goal of teaching and educating people. The power of teachers' motivation directly affects teachers' enthusiasm in teaching and indirectly affects the relationship between the degree of students' social responsibility after employment. In this regard, Chen cultivated students' awareness of social responsibility through moral and rule of law courses and understood the value of social responsibility awareness and the harm of the lack of social responsibility awareness [10]. Using the teacher motivation in different periods to analyze and explore them, the data values obtained are drawn in Table 6.

In Table 6, the survival motivation, responsibility motivation, teacher management system, and social public opinion and expectations are compared and analyzed in different periods. While the data values of various factors under the traditional motivation are all below 55%, compared with the data values of teacher motivation under the innovation, they are all above 60%, which is significantly comparable. According to the statistical method, the data of the two groups were compared, and the difference was significant (*T* < 10.000, *P* < 0.05).

The difference of data values between the two can be more intuitively and clearly compared.  Figure 8 is drawn according to the data values in Table 6.

RETRACTED

As shown in Figure 8, under the comparison of the two kinds of educational motivation, the data value factors of traditional teacher motivation are in a downward trend, while the factors of relatively innovative teacher motivation have a significant upward effect, which has a foundation for improving the quality of education. Good teacher motivation has a great impact on students. Teachers are the beacon of students' life and have a great impact on students' employment, and their cognition of social responsibility is relevant. Under the comprehensive construction and development of Beijing, we should carry out responsibility education for students, so that they can actively and bravely assume their own life responsibilities and better spend a meaningful life. It has important practical significance on the road of life and dare to undertake.

## 8. Discuss

With the continuous development of higher education in China, the number of graduates has increased year by year, and the employment problem has gradually emerged. Nowadays, high-quality talents are in urgent need. Therefore, the cultivation of efficient students and the improvement of their employability are the key tasks at present. Gengfengsong and Wenli pointed out that, to strengthen the employment guidance of college students, teachers should innovate teaching methods, cultivate their ability according to the social employment needs, learn comprehensive knowledge in many aspects, and improve the original limitations, so as to improve their employability [11]. Secondly, Dai proposed that, in order to improve the employability of efficient students, it is important not only to learn theoretical knowledge, but also to practice, and to participate in comprehensive courses. Teachers should establish teaching objectives that are in line with the current development, innovate teaching methods, and improve the trend of difficult employment [12]. In order to further understand the current situation of sollege Students' social responsibility awareness, Hou and Liuhe carried out a questionnaire survey on students in major colleges and universities. The results showed that there were differences in college students' social responsibility awareness, and higher vocational college students of different grades and genders had weak social responsibility awareness. Therefore, they carried out social responsibility awareness education on students to enrich their social responsibility awareness of social practice [13]. Colleges and universities strengthen the cultivation of innovative talents, make use of the influence, exaggeration, and infiltration of the campus environment to imperceptibly educate students, often carry out job competitions and various innovative projects, guide students to correctly grasp the current form of employment, and help students recognize their own advantages and choose employment. We should constantly improve our personal quality in social practice, so as to realize our personal value.

RETRACTED

## 9. Summary

Based on the management efficacy and motivation of teachers, this study studies the impact of college students' academic achievement and postemployment social responsibility cognition, analyzes them through the method of sustainable innovation, and concludes that, under sustainable innovation, teachers' management efficacy and motivation play a key role in students' academic achievement and postemployment social responsibility cognition, and the development of innovative technology has a significant impact on the field of education, making it develop more rapidly. Therefore, the factors of students' academic achievement and social responsibility cognition, teachers' guidance, and education are indispensable. After entering the society, the cognition of social responsibility has been improved, which is conducive to the development of society and better provides the foundation and educational prospects for the field of education. It can better cultivate the ability to serve the society, stimulate the students' sense of responsibility and pursuit of planning and leading social development, and cultivate the sense of responsibility, which can greatly enhance the students' sense of responsibility and mission.

## Figures and Tables

**Figure 1:** The influence of professional titles on teachers' achievement motivation in colleges and universities.

**Figure 2:** Impact of academic qualifications on teachers' professionalism.

**Figure 3:** Analysis of the cycle characteristics of teachers' teaching effectiveness under innovation.

**Figure 4:** Analysis of the formation stage of innovative teachers' teaching ability.

**Figure 5:** Visual analysis of teacher management effectiveness on academic achievement of college students in different periods.

**Figure 6:** Visual analysis of teacher motivation on academic achievement of college students in different periods.

**Figure 7:** Visual analysis of management effectiveness in different periods on students' responsibility cognition after employment.

**Figure 8:** Visual analysis of teachers' motivation on students' social responsibility after employment in different periods.

**Table 1:** Influence of professional titles on teachers' achievement motivation in colleges and universities.

Grouping	Assistant lecturer (%)	Lecturer (%)	Adjunct professor (%)	Professor (%)
Traditional teachers	79	85	88	86

Innovative teachers	88	95	92	94

RETRACTED

**Table 2:** Influence of educational background on teachers' professionalism.

Grouping	Career identity (%)	Professional ethics (%)	Professional knowledge (%)	Professional ability (%)
Junior college education	53	68	65	59

Junior college education	79	81	86	83

Junior college education	95	93	97	92

**Table 3:** Comparison of teaching management effectiveness on academic achievement of college students in different periods.

Grouping	Course learning (%)	Interpersonal communication (%)	Ability development (%)	Academic evaluation (%)
Traditional teachers	40	58	67	43
Innovative teachers	88	85	91	93

**Table 4:** Comparison of teacher motivation on academic achievement of college students in different periods.

Grouping	Achievement motivation (%)	Responsibility motivation (%)	Educational incentives (%)	Pursuit of teaching level (%)
Traditional teachers	48	56	59	47
Innovative teachers	89	94	81	92

**Table 5:** Comparative analysis of management effectiveness in different periods on students' postemployment responsibility cognition.

Grouping	Teacher efficacy (%)	Knowledge management (%)	Social responsibility cognition (%)	Ideals and beliefs (%)
Traditional management effectiveness	39	42	40	35

Innovation management effectiveness	55	61	68	52

**Table 6:** Comparison of teachers' motivation on students' social responsibility after employment in different periods.

Grouping	Survival motivation	Responsible power	Teacher management system	Public opinion and expectation
Traditional teacher motivation	54%	48%	41%	36%
Innovative teacher motivation	70%	67%	60%	59%
*t*	8.234	8.809	9.132	9.526
*P*	0.043	0.041	0.039	0.047

## Data Availability

The data underlying the results presented in the study are available within the manuscript.
